# lncRNA GHET1 Promotes the Progression of Triple-Negative Breast Cancer *via* Regulation of miR-377-3p/GRSF1 Signaling Axis

**DOI:** 10.1155/2022/8366569

**Published:** 2022-04-25

**Authors:** Yu Wang, Chen Li

**Affiliations:** Molecular Testing Center, The First Affiliated Hospital of Jinzhou Medical University, Jinzhou, Liaoning Province 121000, China

## Abstract

**Objective:**

This study is aimed at investigating the role of lncRNA GHET1 in the progression of triple-negative breast cancer (TNBC).

**Methods:**

Tumor tissues and paracancerous tissues (normal) of TNBC patients were collected. Human normal breast cells (MCF10A) and TNBC cells (MDA-MB-468 and HCC1937) were employed for *in vitro* analysis. The expression of lncRNA GHET1, miR-377-3p, and GRSF1 was detected by qRT-PCR. The lncRNA GHET1 and miR-377-3p were overexpressed or knocked down in the TNBC cells, respectively. To determine the specific biological activities of the TNBC cells, MTT, flow cytometry, and wound healing assay were adopted to evaluate the cellular proliferation, apoptosis, and migration abilities, respectively. MMP-9 and MMP-2 protein expression levels were detected as well by Western blot in the cells. The relationship between miR-377-3p and lncRNA GHET1, miR-377-3p, and GRSF1 was validated using dual-luciferase reporter assay.

**Results:**

lncRNA GHET1 was significantly upregulated in the TNBC patients' tissues and the TNBC cell lines. Overexpression of lncRNA GHET1 significantly increased the proliferation and migration ability, but decreased apoptosis in the TNBC cells. Additionally, overexpression of lncRNA GHET1 upregulated both MMP-9 and MMP-2 protein expression levels. Correlation analysis found that miR-377-3p had a positive relationship with GRSF1, but had a negative relationship with lncRNA GHET1. miR-377-3p mimic attenuated the effects of lncRNA GHET1 on cellular proliferation, apoptosis, and migration of the TNBC cells.

**Conclusion:**

lncRNA GHET1 promotes TNBC progression through the miR-377-3p/GRSF1 signaling axis.

## 1. Introduction

Breast cancer (BC) is the most prevalent cancer, becoming the leading cause of cancer death among women worldwide. The American Cancer Society estimated that there were 42,260 BC deaths and 27, 1270 new BC cases in 2019, accounting for about 30% of all female cancer diagnoses [1]. This cancer is divided into five different subgroups based on histological features and molecular biological techniques. Among them, 15%-20% cases belong to triple-negative breast cancer (TNBC). TNBC diagnostic features are negative expression of estrogen receptor (ER), progesterone receptor (PR), and human epidermal growth factor receptor 2 (HER2) [2]. Clinically, it is characterized as high invasiveness and high rates of metastasis, recurrence, and mortality. TNBC frequently metastasizes to internal organs and brain at an early stage; however, it is usually diagnosed at a late stage [3]. The median overall survival of the metastatic TNBC is less than 1 year, whether or not accepting the intensive systemic chemotherapy [4]. Despite significant improvements in BC therapy, the clinical management of TNBC remains challenging compared to the other subtypes because of its aggression and lack of specific targeted therapies [5]. Current clinical treatment options for TNBC are restricted to surgery, radiotherapy, and chemotherapy. Although some studies have shown that TNBC patients are more sensitive to anthracycline-based chemotherapy regimens, the overall survival rate is still low [6]. Therefore, development of specific treatments to prevent and treat BC metastasis is currently a critical aspect of BC research.

Among the new and potentially useful biomarkers, abnormal expression of noncoding RNAs (ncRNAs) has a close relation to TNBC occurrence and progression [7]. Long noncoding RNAs (lncRNAs) are a class of ncRNAs over 200 nucleotides in length, which are believed to be dysregulated in various cancers (breast, ovarian, and others) [8]. Misregulation and mutations of lncRNAs involve tumor pathogenesis. Alterations or mutations of some lncRNA levels could induce tumor growth or metastasis. lncRNAs may appear oncogenic or tumor-suppressive activity. In addition, because of the characteristics of their tissue-specific distribution, lncRNAs may be applied as novel biomarkers for cancer therapy as well [9]. Many dysregulated lncRNAs have been proved to significantly affect TNBC. For example, Zheng et al. found that lncRNA GAS5 could target miR-378a-5p/SUFU to promote TNBC cell apoptosis and regulate the sensitivity of the cancer cells to chemotherapeutic agents [10]. In a study by Wang et al., lncRNAs could regulate TNBC development through the formation of encoded small peptides, such as LINC00908-encoded polypeptide ASRPS, to reduce angiogenesis [11]. In addition, lncRNAs can also control expression levels of their target genes *in cis* or *in trans via* interacting with transcription factors or histone-modifying enzymes. For instance, binding of lncRNA DANCR and RXRA could increase RXRA serine 49/78 phosphorylation and subsequent activate PI3K/Akt signaling, ultimately affecting TNBC cell proliferation [12]. However, there are still many related lncRNAs that have not been explored. It has previously been pointed out that in a hypoxic environment, lncRNA GHET1 can promote TNBC glycolysis, proliferation, and invasion via the Hippo/YAP pathway [13]. However, the role of this lncRNA in TNBC has not been comprehensively elucidated. We therefore attempted to carry out further research.

miRNAs are also a kind of ncRNAs, containing only 20-24 nucleotides [14]. Many of them play a key role in the development and progression of cancers, such as miR-377-3p. Previous study shows that miR-337-3p serves as a tumor suppressor gene in a variety of cancers. Although it has been demonstrated that Linc00339 promotes TNBC progression through the miR-377-3p/HOXC6 signaling pathway [15], the detail mechanism is still uncovered. It is also not allowed to ignore that lncRNAs act as a sponge for miRNAs. Therefore, we try to interrogate what is the relationship between lncRNAs GHET1 and miR-377-3p and what are the effects of them on TNBC, to provide new biomarkers and therapeutic targets of TNBC.

## 2. Materials and Methods

### 2.1. Clinical Samples

20 tumor tissue samples were collected from the patients with luminal A TNBC without any chemotherapy who received surgical section treatment in our hospital between January 2020 and March 2021. The central parts of the tissue were applied as TNBC samples, and the peripheral tissues of the mass were used as normal control tissue. The samples were identified as TNBC tissues by three independent pathologists. This study had obtained informed consent from each patient and an approval from the Ethics Committee of the First Affiliated Hospital of Jinzhou Medical University (KYLL202123).

### 2.2. Cell Culture

TNBC cells (MDA-MB-468 and HCC1937) and human normal breast cells (MCF10A) were provided by the American Type Culture Collection (ATCC, Manassas, VA, USA). The cells were cultured in a complete DMEM containing 10% fetal bovine serum (FBS) (Gibco, EI Paso, Texas, USA), 100 mg/mL penicillin, and 10 mg/mL streptomycin in an incubator with 5% CO_2_ at 37°C.

### 2.3. Cell Transfection

lncRNA GHET1 overexpression plasmid (GHET1), shRNA scramble (sh-NC), lncRNA GHET1 shRNA (sh-GHET1), mimic scramble (NC mimics), miR-377-3p overexpression plasmid (miR-377-3p mimics), miR-377-3p inhibitor (miR-377-3p inhibitor), and inhibitor NC were constructed by GenePharma (Shanghai, China). The plasmids of these constructions were transfected into MDA-MB-468 and HCC1937 cells, respectively, by using Lipofectamine 2000 transfection kit (Sigma-Aldrich, St. Louis, MO, USA). The transfection medium was replaced by complete medium 6 h later, and subsequent experiments were performed after 48 h of the transfection.

### 2.4. qRT-PCR

The nucleus and cytoplasm were extracted by using a Nuclear and Cytoplasmic Extraction Kit (Thermo Fisher Scientific, Waltham, MA, USA). TRizol method (Thermo Fisher Scientific) was employed for RNA extraction from the nucleus, cytoplasm, whole cells, or tissues. The concentration and purity of the extracted RNA was then analyzed by a NanoDrop-based detection. The RNA was then reverse transcribed into cDNA by using a Reverse Transcriptase Kit (Zomanbio, Beijing, China). lncRNA GHET1, miR-377-3p, or GRSF1 was amplified with the cDNA by using a SYBR GREEN kit (TaKaRa, Tokyo, Japan). The primers of the lncRNAs GHET1, miR-377-3p, and GRSF1 are listed in Table 1. Six replicates were set up for each experiment. U6 or GAPDH was applied as internal reference controls. Quantification of the target gene relative expression was analyzed by the 2^-*ΔΔ*Ct^ method.

### 2.5. MTT Assay

MDA-MB-468 or HCC1937 cells were seeded in 96-well plates (5000 cells/well) for 24 h. The cells were stained with 20 *μ*L of 5 mmol/L MTT for 4 h in a 37°C incubator. After that, 150 *μ*L of DMSO was added to melt the cells for 15 min. Finally, the viability rate was detected by OD 450 nm measurement.

### 2.6. Apoptosis Assay

The Annexin V-FITC/PI Apoptosis Detection Kit (Yeasen, Shanghai, China) was employed to do the apoptosis assay. MDA-MB-468 cells or HCC1937 cells to be detected were collected into a centrifuge tube, twice rinsed with precooled sterile PBS, and adjusted to 5 × 10^5^ cells/mL. Subsequently, 200 *μ*L of the cell suspension, 10 *μ*L of Annexin V-FITC, and 10 *μ*L of 20 mg/L PI solution (all from the kit) were mixed and incubated at avoiding light condition at room temperature for 10 min, followed by dilution with 500 *μ*L of the PBS. The apoptotic rate was detected by a FACSCalibur flow cytometer (BD Biosciences, CA, USA).

### 2.7. Wound Healing Assay

Treated cells were seeded into 6-well plates and cultured until confluence. A 10 *μ*L sterile tip was applied to scratch the cells to create a wound field. After removing the cellular debris and detached cells by PBS, fresh serum-free medium was added for 24 h culture. The migrated cells on the scratched area were photographed under an inverted microscope. ImageJ software was used to calculate the migrated area from the original scratched wound area.

### 2.8. Western Blotting

The protein concentration of the cellular or tissue lysate was detected with a BCA Protein Assay Kit (Beyotime, Shanghai, China). Each 20 *μ*g of the samples to be detected was boiled in 1x Loading Buffer (Beyotime) and cooled on an ice box, loaded and separated on a SDS-PAGE, and transferred to a PVDF membrane for 1 h. The membrane was then blocked with 5% nonfat dry milk for 1 h, incubated with corresponding primary antibody overnight at 4°C, triplicate rinsed with 1x TBS-T buffer (Beyotime), continue reacted with corresponding secondary antibody for 1 h, and triplicate washed with TBS-T again. For protein development, Chemiluminescence Reagents (Beyotime) were dropped on the membrane for 1 min. The acquisition of images was completed using a Gel Imaging System (Thermo Fisher, Waltham, MA, USA). Densitometry of the target protein bands was analyzed by the ImageJ software. GAPDH was applied as an internal reference to calculate the relative protein expression.

### 2.9. Dual-Luciferase Reporter Assay

293T cells (ATCC) were transfected with NC mimics/miR-377-3p mimics and dual-luciferase reporter vectors of lncRNA GHET1 wild type (WT-GHET1)/mutant (MUT-GHET1) or GRSF1 wild type (WT-GRSF1)/mutant (MUT-GRSF1), respectively. Firefly and Renilla luciferase activities were measured 48 h later using a dual-luciferase reporter assay system (CAS: E1910, Promega, Madison, Wisconsin, USA). The luciferase activity was recorded with a GloMax 96 Microplate Fluorometer (Promega).

### 2.10. Statistical Analysis

SPSS 26.0 was used for statistical analysis. One-way analysis of variance and independent sample *t*-test analysis were employed for comparison among multiple groups and between two groups, respectively. The results were expressed as mean ± standard deviation (SD). Further, Pearson correlation was used to analyze the expression correlation between two parameters in tissue samples. *P* < 0.05 served as the cutoff value of a significant difference.

## 3. Results

### 3.1. The Expression of lncRNA GHET1 Is Significantly Upregulated in TNBC

According to qRT-PCR results regarding lncRNA GHET1 expression in TNBC, we found that the lncRNA was significantly increased in the TNBC tissue (Figure 1(a)), as well as in HCC1937 and MDA-MB-468 cells (Figure 1(b)). At the cellular level, lncRNA GHET1 showed the highest expression at TNBC cell HCC1937. These results suggested that lncRNA GHET1 might play a role in TNBC oncogenes.

### 3.2. lncRNA GHET1 Promotes the Malignant Process of TNBC Cells

To validate the role of lncRNA GHET1 in TNBC development, the lncRNA was overexpressed in MDA-MB-468 cells and knocked down in HCC1937. The efficacy of the overexpression and knockdown was checked by qRT-PCR (Figure 2(a)). MTT assay for cell proliferation, flow cytometry for apoptosis, and wound healing assay for migration ability found that lncRNA GHET1 overexpression has an oncogenic activity to remarkably increase the cellular proliferation and migration and obviously decrease the apoptosis, while knockdown of the lncRNA GHET1 caused the opposite changes (Figures 2(b)–2(e)). Further examination of the protein expression of matrix metalloproteinases 9 (MMP-9) and 2 (MMP-2) showed that the protein expression levels of MMP-9 and MMP-2 were significantly increased after overexpression of the lncRNA GHET1 in the cells, but decreased after its knockdown (Figure 2(f)), indicating that both MMP-9 and MMP-2 were closely related to tumor migration. The results above indicated that lncRNA GHET1 was involved in the oncogenes of TNBC.

### 3.3. lncRNA GHET1 Acts as a miR-377-3p Sponge in TNBC

The detailed mechanism by which lncRNA GHET1 affects TNBC progression was further investigated. Analysis of subcellular distribution of the lncRNA GHET1 showed that it was mainly distributed in the cytoplasm (Figure 3(a)). Interestingly, ENCORI (https://starbase.sysu.edu.cn/) prediction revealed a binding site of lncRNA GHET1 and miR-377-3p. It was verified by dual-luciferase assay that miR-377-3p overexpression reduced the fluorescence intensity of lncRNA WT-GHET1 without affecting that of MUT-GHET1-MUT (Figure 3(b)).

Noticeably, miR-377-3p level was significantly decreased in TNBC tissues (Figure 3(c)). Subsequent detection revealed that overexpression of lncRNA GHET1 declined the miR-377-3p level. However, knockdown of lncRNA GHET1 significantly elevated the miR-377-3p level (Figure 3(d)). Correlation analysis showed a negative correlation between the lncRNA GHET1 and miR-377-3p (Figure 3(e)). Collectively, lncRNA GHET1 targeted to miR-377-3p in TNBC.

### 3.4. Knockdown of miR-377-3p Reversed the Effect of lncRNA GHET1 Knockdown on TNBC Cells

To validate the role of the interaction of lncRNA GHET1 and miR-377-3p in TNBC, we performed rescue experiments. TNBC cells were treated with simultaneous overexpression or knockdown of either lncRNAs GHET1 or miR-377-3p. The biological performance of cells was then measured. According to the results, lncRNA GHET1 mimics (GHFT1) significantly upregulated GRSF1 protein expression, cellular proliferation, and migration, but decreased cellular apoptosis in the MDA-MB-468 cells. However, such alterations were obviously reversed by GHET1+miR-377-3p mimic overexpression in the HCC1937 cells. Furthermore, sh-lncRNA GHET significantly reduced GRSF1 protein expression and cellular proliferation and migration, but promoted apoptosis. Interestingly, transfection with both sh-lncRNA GHET and miR-377-3p inhibitor successfully reversed the alteration patterns induced by sh-GHFT1 (Figures 4(a)–4(d)). Collectively, knockdown of miR-377-3p restored the lncRNA GHET knockdown-induced inhibitory effect on the malignant progression of TNBC cells.

### 3.5. GRSF1 Was a Target Gene of miR-377-3p

To further investigate the antioncogenic mechanism of miR-377-3p, we used the TargetScan program (http://www.targetscan.org/vert_72/) to predict the target genes of miR-377-3p, which found an interaction site between miR-377-3p and GRSF1 (Figure 5(a)). Further, miR-377-3p overexpression significantly inhibited the fluorescence intensity of WT-GRSF1. However, it did not affect MUT-GRSF1 fluorescence intensity by the dual-luciferase reporter assay (Figure 5(a)), demonstrating that there was an interaction between miR-377-3p and GRSF1.

GRSF1 expression was found to be significantly increased in TNBC tissues by qRT-PCR (Figure 5(b)). Both the mRNA and protein expression of GRSF1 was upregulated by miR-377-3p inhibitor. However, miR-377-3p mimic obviously decreased the expression levels of GRSF1 in the TNBC cells (Figures 5(c)–5(e)). Correlation analysis also showed a negative correlation between GRSF1 and miR-377-3p (Figure 5(f)).

The regulation of GRSF1 by lncRNA GHET1 was subsequently investigated as well. The results showed that lncRNA GHET1 mimic significantly increased GRSF1 expression in the TNBC cells, while knockdown of lncRNA GHET1 led to a decreased expression of GRSF1 (Figure 5(g)). Correlation analysis also indicated a positive relationship between GRSF1 and lncRNA GHET1 (Figure 5(h)). Collectively, GRSF1 was a target gene of miR-377-3p, and lncRNA GHET1 could regulate miR-377-3p/GRSF1 to affect the process of TNBC.

## 4. Discussion

TNBC is an aggressive subtype of BC, and its progression is attributed to a variety of oncogenes and tumor suppressor genes. A full understanding of molecular events and identification of critical biomarkers can improve the efficacy of TNBC therapy [16]. In recent years, increasing evidence strongly supports the involvement of lncRNAs in the pathogenesis and progression of human cancers [17]. In order to develop new cancer treatments, the functions and mechanisms of lncRNAs require further investigation. lncRNA GHET1 has been shown to be a key regulatory molecule in the development of many cancers. Zhu et al. found that lncRNA GHET1 also enhanced the proliferation of prostate cancer cells through activation of HIF-1*α*/Notch-1 signaling by binding to KLF2 [18]. It is worth noting that inhibition of lncRNA GHET1 could downregulate the expression of EGFR protein and inhibit PI3K/AKT signaling activity, thereby inhibiting the cellular activity of BC [19]. Consistent with previous studies, our study showed that lncRNA GHET1 was significantly upregulated in TNBC tissues and cells. High expression of the lncRNA GHET1 significantly promoted cell proliferation and migration and inhibited apoptosis. These findings suggest that lncRNA GHET1 plays a key role in the development of TNBC.

Similar to other cancers, the therapy for BC includes surgical resection, chemotherapy, radiotherapy, and targeted therapy. Endocrine therapy could also be applied to common BC. Although the benefits of chemotherapy are limited, TNBC is sensitive to it and still the standard treatment. Only a small partial of TNBC patients respond to targeted immunosuppressive sites or poly-ADP-ribose polymerase (PARP) inhibitors. However, they often develop drug resistance and even recurrence. There are few other options for TNBC therapy [20]. The finding of this study that lncRNA GHET1 regulates TNBC via the miR-377-3p/GRSF1 pathway undoubtedly provides a new clue for the treatment of TNBC.

It is now generally recognized that the expression of lncRNAs can be used as a signal of a specific cell state or a measure of active cellular processes. Hence, this kind of biomarkers can provide prognostic value for cancer and even provide treatment options for cancer patients [21]. Recent studies have shown that lncRNAs can regulate gene expression at different levels, including chromatin modification and transcriptional and posttranscriptional regulation [22]. They can act as miRNA and compete with miRNA-targeted mRNAs, thereby affecting miRNA-mediated gene regulation [23]. This crosstalk forms a complex posttranscriptional regulatory network that includes mRNAs and lncRNAs and is called competitive endogenous RNA (ceRNA) network. The ceRNA-mediated regulatory mechanism is an important pathway for posttranscriptional regulation by lncRNAs in TNBC. The ceRNA regulatory network can help us understand the potential characteristics of biological functions and pathological roles of lncRNAs in TNBC development and progression [24]. In this study, lncRNA GHET1 was found to directly target miR-377-3p as an ecRNA. Previously, it has been shown that miR-377-3p acts as a tumor suppressor in many types of cancers. For example, it inhibited the development and progression of esophageal cancer by targeting CD133 and VEGF [25] and inhibited gastric cell proliferation and metastasis by suppressing VEGFA expression [26]. Moreover, miR-377-3p is an important component of the ceRNA network mediated by lncRNAs during cancer development. Existing studies reported that LINC00339 promoted gastric cancer progression by inhibiting miR-377-3p to increase DCP1A expression [27]. lncRNA SNHG4 promoted osteosarcoma proliferation and migration by sponging miR-377-3p [28]. In this study, we also found that miR-377-3p could reverse the effects induced by overexpression of lncRNA GHET1 on TNBC cells, demonstrating the joint involvement of lncRNA GHET1 and miR-377-3p in TNBC development.

GRSF1 is a mitochondrial RNA-binding protein, a guanine-rich sequence factor, and a component of the mitochondrial RNA particle, large ribonucleoprotein (RNP) structure [29]. Previous studies have pointed out that GRSF1 is required to maintain mitochondrial function and that loss of GRSF1 triggers DNA damage and impairs cell proliferation [30]. During the development of cancer, GRSF1 expression is significantly increased, and high expression of GRSF1 predicts a poor prognosis [31]. In this study, we found that GRSF1 was a target gene of miR-377-3p, and it was significantly elevated in TNBC tissue. To determine the role of lncRNA GHET1/miR-377-3p/GRSF1 in TNBC, we simultaneously knocked down or overexpressed lncRNAs GHET1 and miR-377-3p, and correspondingly, GRSF1 expression was affected and biological performance of TNBC cell was also influenced. Such findings suggest that the lncRNA GHET1/miR-377-3p/GRSF1 network plays a critical role in TNBC development.

MMPs belong to zinc endopeptidases which act as critical factors for extracellular matrix (ECM) degeneration [32]. MMPs play crucial roles in many pathological and physiological issues, including inflammation, embryonic development, wound healing, tumor metastasis, and invasion [33]. In cancer, elevation of MMP-2 and MMP-9 causes ECM degradation, resulting in tumor invasion and metastasis [34]. In addition, MMP-2 and MMP-9 also involve tumor growth through regulation of cellular proliferation, apoptosis, and angiogenesis [35–37]. Upregulation of MMP-2 and MMP-9 by lncRNA GHET1 clearly exhibits the oncogenic mechanism of the lncRNA GHET1 *via* MMP-2 and MMP-9 regulation.

## 5. Conclusions

In summary, lncRNA GHET1 enhances TNBC cell proliferation and migration ability and reduces apoptosis by regulating the miR-377-3p/GRSF1 pathway, thus playing a cancer-promoting role in TNBC. These results suggest that lncRNA GHET1/miR-377-3p/GRSF1 may be a potential prognostic marker and therapeutic target of TNBC.

## Figures and Tables

**Figure 1:** lncRNA GHET1 expression is increased in TNBC. qRT-PCR-based measurement of lncRNA GHET1 expression in tissues ((a) ^∗∗^*P* < 0.01*vs*. the normal group) and in indicated cells ((b) ^∗∗^*P* < 0.01*vs.* the MCF10A group).

**Figure 2:** Oncogenic activity of lncRNA GHET1 in TNBC cells. (a) lncRNA GHET1 expression was analyzed by qRT-PCR in the lncRNA GHET1 overexpressed (GHET1) MDA-MB-168 and knocked down (sh-GHFT1) HCC1937 cells. (b) Cellular proliferation was detected by MTT assay in the indicated cells. Cellular apoptosis was analyzed by flow cytometry in the (c) MDA-MB-468 and (d) HCC1937 cells. (e) Cellular migration was evaluated by wound healing assay in the indicated cells. (f) Protein expression levels of MMP-9 and MMP-2 were detected by Western blot in the indicated cells, ^∗∗^*P* < 0.01 vs. the vector/sh-NC group. Each data came from independent triplicate assays.

**Figure 3:** Relationship between lncRNA GHET1 and miR-377-3p in TNBC. (a) Cellular distribution of lncRNA GHET1 was analyzed by qRT-PCR-based measurement in the nucleus (blue) or cytoplasm (grey). ^∗∗^*P* < 0.01*vs*. the cytoplasm group. (b) The relationship between lncRNA GHET1 and miR-377-3p was analyzed by dual-luciferase reporter gene assay in the indicated groups. ^∗∗^*P* < 0.01*vs*. the NC mimic group. miR-377-3p expression was detected by qRT-PCR in the TNBE tissues; peripheral tissues of the mass were used as (c) negative control (normal) and (d) indicated TNBC cells. ^∗∗^*P* < 0.01*vs*. the normal group *vs.* the vector/sh-NC group. (e) The correlation between lncRNA GHET1 and miR-377-3p expression was analyzed by the Pearson correlation method in the TNBC tissues. Each data in (a–d) represented the average of three independent assays.

**Figure 4:** miR-377-3p inhibitor reversed the lncRNA GHET1 mimic-induced bioactivities in TNBC cells. GRSF1 (a) protein expression, (b) cellular proliferation, (c) cellular apoptosis, and (d) cellular migration were detected by (a) Western blot, (b) MTT assay, (c) flow cytometry, and (d) wound healing assay, respectively, in the indicated cells. ^∗∗^*P* < 0.01*vs*. vector/sh-NC, ^##^*P* < 0.01*vs*. GHET1/sh-GHET1. Each data was the average of three independent assays.

**Figure 5:** GRSF1 is a downstream target of miR-377-3p. (a) Target gene of miR-377-3p was predicted by the TargetScan database (up panel). Interaction between miR-377-3p and GRSF1 was analyzed by dual-luciferase reporter gene, ^∗∗^*P* < 0.01*vs*. NC mimics. (b) GRSF1 expression was detected by qRT-PCR in TBNC tissues, ^∗∗^*P* < 0.01 vs. the normal group. (c) miR-377-3p expression was detected by qRT-PCR in the indicated TNBC cells. (d) GRSF1 protein expression was detected by Western blotting in the indicated TNBC cells. (e) GRSF1 mRNA expression was detected by qRT-PCR in the miR-377-3p mimic- or inhibitor-transfected TNBC cells, ^∗∗^*P* < 0.01*vs*. NC mimics/NC inhibitor. (f) Correlation between miR-377-3p and lncRNAGRSF1 in TNBC tissues was analyzed by Pearson correlation. (g) qRT-PCR was used to detect GRSF1 expression in the TNBC cells overexpressed or knocked down lncRNA GHET1, ^∗∗^*P* < 0.01 vs. the vector/sh-NC group. (h) Correlation between GRSF1 and lncRNA GHET1 in TNBC tissues was analyzed by Pearson correlation analysis. Each data was the average of three independent assays.

**Table 1:** Primer sequences.

RNA	Sequences (5′ to 3′)
lncRNA GHET1	F: CAACAAAGCAGGTAAACATTGG
	R: GCAAAGGCAGAGTGAAAGGT
miR-377-3p	F: ATCACACAAAGGCAACTTTTGT
	R: GGTGCAGGGTCCGAGGTAT
GRSF1	F: TGGAGTCAGAGCAGGATGTGCA
	R: GGCGAAGATTTGACCTGCAAGC
GAPDH	F: GTCTCCTCTGACTTCAACAGCG
	R: ACCACCCTGTTGCTGTAGCCAA
U6	F: CTCGCTTCGGCAGCACA-3′
	F: AACGCTTCACGAATT TGCGT-3′

F: forward primer; R: reverse primer.

## Data Availability

The data used to support the findings of this study are available from the corresponding author upon request.
